# Alternative Water Resources Selection to Supply Drinking Water in Flood Disasters by Multicriteria Decision-Making Techniques (DANP and VIKOR)

**DOI:** 10.1155/2022/5445786

**Published:** 2022-06-13

**Authors:** Aman Allah Zamani, Hamid Reza Abbasi, Vali Alipour, Mahmoudreza Peyravi, Payam Shojaei, Ali Goli, Leila Mohammadinia

**Affiliations:** ^1^Department of Health in Disasters and Emergencies, Health Human Resources Research Center, School of Management and Medical Informatics, Shiraz University of Medical Sciences, Shiraz, Iran; ^2^Trauma Research Center, Shahid Rajaee (Emtiaz) Trauma Hospital, Shiraz University of Medical Sciences, Shiraz, Iran; ^3^Environmental Health Engineering, School of Health, Hormozgan University of Medical Sciences, Bandar Abbas, Iran; ^4^Department of Health in Disasters and Emergencies, School of Management and Medical Informatics, Shiraz University of Medical Sciences, Shiraz, Iran; ^5^Department of Management, Shiraz University, Shiraz, Iran; ^6^Department of Sociology & Social Planning, Shiraz University, Shiraz, Iran; ^7^Department of Health Policy and Management, School of Management and Medical Informatics, Tabriz University of Medical Sciences, Tabriz, Iran

## Abstract

**Background:**

Emergency is generally caused by natural disaster and infectious disease outbreaks, or it is man-made. Floods are natural phenomena that generally appear in multiple parts of the world. Flooding is one of the most destructive naturally occurring environmental hazards and can cause public, infrastructural, and environmental damage. The purpose of this study is to select alternative water resources for supplying Bandar Abbas in flood disasters by multicriteria decision-making techniques.

**Methods:**

Information required includes possible water resources alternative for flood, quantitative and qualitative characteristics of the water resources, climatic circumstances, and demographic information used in organizations data and previous studies. After selecting and proposing water resources alternative for Bandar Abbas in flood, the subcriteria were weighed applying DANP (DEMATEL-ANP) techniques and water resources were prioritized with the VIKOR technique. According to the network structure and internal and external dependence of the criteria and subcriteria, the advantages of DANP in calculating weights have been used to adapt to more real-world problems. The VIKOR technique was developed for multicriteria optimization of complex systems.

**Results:**

After reviewing and extracting the criteria from various studies, 9 main criteria and 44 subcriteria were defined to select water resources in disasters and emergencies. According to field studies and related organizations' information, the proposed water resources for Bandar Abbas to use in flood disasters include humidity, sea (Persian Gulf), Sarkhoon plain, and wastewater treatment plant of Bandar Abbas.

**Conclusion:**

Results showed that the optimal water resources for Bandar Abbas in flood disasters are the sea and wastewater treatment plant effluent (after advanced treatment). The study proposed appropriate model to select optimal water resources for various natural disasters in different geographical areas. This model can help officials and decision-makers to plan for drinking water supply from disaster-prone areas before disasters occur.

## 1. Introduction

An emergency means a condition or status where the people's ability decreases and they cannot buck up their ordinary livelihoods because of losses or dangers to their health and life. Emergency is generally caused by natural disaster (earthquake, flood, and drought) and infectious disease outbreaks (coronavirus, Ebola, and influenza pandemic), or it is man-made (chemical leakage) [1]. Floods are natural phenomena that generally appear in multiple parts of the world. However, the event of flood incidents is expected to increase universally in the future, as climatic changes will cause more severe rainfall in some regions [2]. Flooding is one of the most destructive naturally occurring environmental hazards and can cause public, infrastructural, and environmental damage [3].

Numerous people were affected by a shortage of clean water for drinking and sanitation during the flood. In addition, tap water turbidity (containing sediment) was found at or around the regions affected by the flood. This turbidity increased during the flood and made the water unfit for human consumption. Floods can result in the mixing of clean water with unsafe water. Tap and drinking water can become contaminated by flood at the resources where the water is supplied or via the distribution systems. Following such contamination, the incidence of certain diseases such as cholera, typhoid fever, leptospirosis, and hepatitis A can rise and affect enormous numbers of individuals [4].

Iran is among the ten most disaster-prone countries in the world. Of 43 known global events, 34 events have occurred in Iran. Statistics showed that 90% of the Iranian population is exposed to earthquakes and floods [5]. In 100 years between 1920 and 2020 in Iran, 243 cases of disasters triggered by natural hazards occurred. The cause of 37.4% (91 events) was flood. There were 157,274 deaths during this period, of which 5.1% (8048 deaths) were due to floods. The economic damage during this period was estimated at approximately 50.6 billion dollars, of which 41.59% (21 billion dollars) was due to floods. More than 55 million people were affected by natural disasters during this period, of which 26.03% (more than 14 million people) were due to floods [6].

In disasters, available water resources for sanitary purposes, drinking, and cooking are very limited. Therefore, it is necessary to consider the appropriate volume of water for sanitary purposes to prevent the occurrence of diseases caused by dehydration [7]. In the past, drinking water supply in the disaster areas was mainly in the form of bottled water or transfer by water tankers from different areas [8], and, due to the possibility of a long recovery phase, the need for safe water in the disaster area is not fully met, and this causes health problems in the area. Using water resources in the affected area is more practical and sustainable [9].

The study area of Bandar Abbas is one of the most important cities in the south of Iran and the political center of Hormozgan province. In the 2016 census, its population was 526848 people [10]. Bandar Abbas is sea coastal and has hot and humid weather, long hot summers, and short mild winters. Due to the economic and political importance of the city, the natural hazards that threaten it, and the lack of proper planning for water supply in emergencies, Bandar Abbas was selected as the study area.

Lack of proper planning for areas with different geographical and cultural conditions, no consideration of further criteria and subcriteria aspects for selecting water resources, and lack of attention to the water resources capacity and availability in a disaster-prone area are the challenges.

This study aims to determine the main criteria and subcriteria for selecting water resources in disasters for drinking water supply and then weighing the selected criteria for flood disasters using a combination of Decision-Making Trial and Evaluation Laboratory (DEMATEL) and Analytic Network Process (ANP). Also, according to the characteristics and geographical features of the study area, the available water resources for water supply in floods are determined. The identified water resources are prioritized using the criteria weight with Vlse Kriterijumsk Optimizacija Kompromisno Resenje (VIKOR) technique. Finally, the most suitable water resource available is selected.

### 1.1. Literature Review

Qu et al. used fuzzy TOPSIS techniques to select the best water technologies for different emergency water supply scenarios. The results show that, in the scenarios related to the source of clean and fresh water, expected minimum level of treatment, and the source of brackish water, the use of technology with maximum effective removal of pollutants is essential. Also, in the scenario related to the source of saline water and turbidity of membrane technologies, in particular Ultrafiltration plays the most significant role in the emergency response of drinking water [11].

Pagsuyoin et al. proposed a multicriteria decision-making approach to evaluate and select appropriate point-of-use water treatment technology options for low-income communities. The results showed that water treatment with *Moringa oleifera* and ceramic filters are the best treatment options, while chlorination is the least desirable. The most important criteria for selecting water treatment methods are initial costs, water by-products, production rate, and energy consumption [12].

Sadeghi Yekta et al. used hierarchical distance-based fuzzy multicriteria group decision-making as a tool to evaluate the drinking water supply systems of Qom, a semiarid city in central Iran. The results showed that the “general desalination system” was the most suitable alternative to meet the drinking water need in a semiarid region. Bottled drinking water was the second acceptable option [13].

Malek Mohammadi et al. applied the hierarchical analysis process to plan water resources in emergencies for the city of Pardis near the municipality of Tehran in Iran, which is very vulnerable to earthquakes and floods. The study suggests mobile water treatment and well drilling as water resources in emergencies [14].

Saiful et al. used forward osmosis membranes with chitosan bags to treat seawater and dirty water in emergencies. Results showed that the chitosan bag can be an alternative solution for drinking water supply in emergencies [15].

Amorim used a multicriteria method of the fuzzy hierarchical analysis process to rank the three main alternatives (rainwater harvesting system, grey water recycling system, and water-saving devices) in low-income resorts in Brazil. The main results show that the appropriate option for integrated urban water management is water-saving devices [16].

Santos examined the implementation and application of different point-of-use (POU) water treatment options. Evaluation of each alternative was done using a set of criteria based on environmental sustainability, technological performance, financial sustainability, and social acceptability. Analytic Hierarchy Process (AHP) and TOPSIS techniques were applied to weight and rank the POU options. Results showed that water treatment with *Moringa oleifera* and membrane filtration technologies are the most suitable option at the POU (point-of-use) site [17].

Ma et al. proposed a new strategy to address multicriteria group decision-making problems named the complex Pythagorean fuzzy VIKOR (CPF-VIKOR) method. This method manages a great deal of vagueness and hesitation which are often present in human decisions. The CPF-VIKOR method allows the linguistic terms to express individual opinions of experts about the performance of alternatives and the weights of the criteria. They combined the individual judgments of experts with the help of a complex Pythagorean fuzzy weighted averaging operator. Further, they computed the ranking measure with the help of group utility and regret measures by adjusting the weight of the strategy of maximum group utility within the unit interval [18].

Komazec et al. proposed a hybrid model based on the Analytic Hierarchy Process (AHP) and multicriteria compromised ranking (VIKOR), as applied through the selection of the best medium for informing the population in situations of emergency. The AHP method is used to determine criteria weight coefficients, while the VIKOR method is applied to find the best media through making a selection among numerous alternatives options [19].

Akram et al. presented a multiskilled and high potential multicriteria group decision-making (MCGDM) technique, namely, complex spherical fuzzy VIKOR (CSF-VIKOR) method, using the grounds of VIKOR method and motivation of CSF model which is adequate to deal with two-dimensional data; the working rule of the proposed technique emphasizes proposing a compromised solution depending upon two focal properties, namely, group utility and individual regret of an opponent. The authors sorted the alternatives via the ranking measure by dint of ascending order and validated the precision and veracity of the proposed strategy by comparing the results with the spherical fuzzy VIKOR (SF-VIKOR) method [20].

Pribićević et al. developed a multicriteria method for objectively processing fuzzy linguistic information by comparing possible pairs of criteria. This technique was obtained through the development of the fuzzy DEMATEL-D method. Combining D-numbers with trapezoidal fuzzy language variables (LVs) allows additional processing of the uncertainties and ambiguities that exist in the preferences of experts when comparing criteria with each other. In addition, the fuzzy DEMATEL-D method has a unique reasoning algorithm that allows logical processing of uncertainties when using fuzzy linguistic expressions for pairwise comparisons of criteria. The fuzzy DEMATEL-D method provides a basic uncertainty management framework that is logical and concise [21].

Akram et al. designed a new multifeature group decision-making method called the trapezoidal bipolar fuzzy VIKOR method. This includes a convenient redesign of the VIKOR approach to use information with bipolar settings. Bipolar fuzzy sets (and numbers) create a symmetrical exchange between the two judgmental components of human thought. Agents obtain vague information in the form of linguistic variables that are parameterized by trapezoidal bipolar fuzzy numbers [22].

Akram et al. proposed two novel modified techniques, namely, Pythagorean fuzzy hybrid Order of Preference by Similarity to an Ideal Solution (PFH-TOPSIS) method and Pythagorean fuzzy hybrid ELimination and Choice Translating REality I (PFH-ELECTRE I) method, in order to measure risk rankings in failure modes and effects analysis (FMEA). These methods are designed to overcome the flaws and shortcomings of traditional crisp risk priority numbers and fuzzy FMEA techniques in risk rankings. The PFH-TOPSIS approach computes the distances of failure modes from the Pythagorean fuzzy positive ideal solution and Pythagorean fuzzy negative ideal solution. To evaluate failure modes, the PFH-ELECTRE I approach produces Pythagorean fuzzy concordance and Pythagorean fuzzy discordance matrices [23].

## 2. Materials and Methods

Figure 1 shows the flow diagram of the study method. The main criteria and subcriteria for water resources selection in disasters and emergencies are extracted from reviewing previous studies [24]. Information required includes possible water resources alternative for flood, quantitative and qualitative characteristics of the water resources, climatic circumstances, and demographic information. Demographic and climatic circumstances, respectively, were gathered from the National Statistics Center of Iran, Meteorological Organization. Also, alternative water resources for use in floods information was gathered from Water and Wastewater Company, Regional Water Organization, Environmental Protection Organization, and Health Center of Hormozgan. In the case of lack of information, previous studies' data were utilization.

### 2.1. Weighing Subcriteria

A combination of the ANP and DEMATEL techniques utilizing Excel software for weighing the criteria was used. ANP technique controls the dependence within (Internal) and between (external) different clusters [25]. Its purpose was to solve the problems of interdependence and feedback between criteria and options in the real world. The DEMATEL technique allows us to understand the structure of the impact between the criteria and try discovering problems that can improve. DEMATEL with ANP technique was used to find the most important criteria that help to improve performance. The DEMATEL technique is applied to determine the effect of these criteria and their use to normalize the weightless supermatrix in ANP to mimic the real-world situation [26].

### 2.2. DANP Technique Steps

**Step 1 .**

Specify the direct connection matrix

Evaluation of relationships between criteria (effect of one on another criterion) based on the views of experts utilizing a rating scope from 0 to 4 was done, in which 0 means ineffectiveness, 1 means low, 2 means moderate, 3 means lot of, and 4 means too many impacts. Experts specify the effect of one criterion on another. In this step, we calculate the average view of experts (in this study, 8 experts).

(1) $$\begin{array}{c} D=\left[\begin{array}{ccccc} d_{c}^{11} & \ldots & d_{c}^{1j} & \ldots & d_{c}^{1n}\\ \vdots & \; & \vdots & \; & \vdots \\ d_{c}^{i1} & \ldots & d_{c}^{ij} & \ldots & d_{c}^{in}\\ \vdots & \; & \vdots & \; & \vdots \\ d_{c}^{n1} & \ldots & d_{c}^{nj} & \ldots & d_{c}^{nn} \end{array}\right]. \end{array}$$

**Step 2 .**

Normalize the direct connection matrix

The direct correlation matrix *D* is normalized utilizing the following equation, and matrix *N* is got:

(2) $$\begin{array}{c} N=VD,\\ V=\min\left\{\frac{1}{\max i\sum_{j=1}^{n}d_{c}^{ij}},\frac{1}{\max j\sum_{i=1}^{n}d_{c}^{ij}}\right\},\;i,\;j\in \left\{1,2,\ldots ,n\right\}. \end{array}$$

**Step 3 .**

Calculate the full criteria communication matrix

Once matrix *D* is normalized and matrix *N* is acquired, the communication matrix via the following equation is gained. In this relation, *I* represents the unit matrix.

(3) $$\begin{array}{c} Tc=N+N^{2}+\ldots +N^{h}=N{\left(I-N\right)}^{-1},\;\text{when}\underset{h⟶\infty }{\lim}N^{h}. \end{array}$$

**Step 4 .**

Calculate the complete correlation matrix of the dimensions as well as the intensity and effect direction

First, the TD matrix must be extracted from the complete correlation matrix of the *T*_*c*_ criteria. Thus, each TD matrix component is calculated from the average of the objects as*T*_C_

(4) $$\begin{array}{c} T_{c}=\begin{array}{c} D_{1}\\ \vdots \\ \vdots \\ \vdots \\ D_{i}\\ \vdots \\ \vdots \\ \vdots \\ D_{n}\\ C_{11}\\ C_{12}\\ C_{1_{m_{1}}}\\ \vdots \\ C_{i_{1}}\\ C_{i_{2}}\\ C_{i_{mi}}\\ \vdots \\ C_{n_{1}}\\ C_{n_{2}}\\ C_{nm_{m}} \end{array}\left[\begin{array}{ccccc} T_{c}^{11} & \ldots & T_{c}^{1j} & \ldots & T_{c}^{1n}\\ \vdots & \; & \vdots & \; & \vdots \\ \vdots & \; & \vdots & \; & \vdots \\ \vdots & \; & \vdots & \; & \vdots \\ T_{c}^{i1} & \ldots & T_{c}^{ij} & \ldots & T_{c}^{in}\\ \vdots & \; & \vdots & \; & \vdots \\ \vdots & \; & \vdots & \; & \vdots \\ \vdots & \; & \vdots & \; & \vdots \\ T_{c}^{n1} & \ldots & T_{c}^{nj} & \ldots & T_{c}^{nn} \end{array}\right],\\ T_{D}=\left[\begin{array}{ccc} t_{D}^{11} & \cdots & t_{D}^{1n}\\ \vdots & \ddots & \vdots \\ t_{D}^{n1} & \cdots & t_{D}^{nn} \end{array}\right]. \end{array}$$

The sum of the rows and columns of the complete relational matrix of the dimensions and criteria is calculated separately according to the following equation:

(5) $$\begin{array}{c} T=\left[t_{g}\right],\;i,\;j\in \left\{1,2,\ldots ,n\right\},\\ r={\left[r_{i}\right]}_{n\times 1=}{\left[\overset{n}{\underset{j=1}{\sum }}t_{ij}\right]}_{n\times 1},\\ c={\left[c_{j}\right]}_{1\times n=}{\left[\overset{n}{\underset{j=1}{\sum }}t_{ij}\right]}_{1\times n}. \end{array}$$

The index *r*_*i*_ represents the sum of rows *I* and *c*_*j*_ represents the sum of columns *j* (according to *T*_*C*_^*ij*^ corresponding to the desired dimension).

**Step 5 .**

Normalization of full-dimensional relation matrix (*T*_*D*_^∝^)

The sum of each row is calculated and each element is divided by the sum of the corresponding row elements, and then the row and column of the resulting matrix are replaced. The fully normalized communication matrix *T*_*D*_ is shown as *T*_*D*_^∝^.

(6) $$\begin{array}{c} T_{D}=\left[\begin{array}{ccccc} t_{11}^{D_{11}} & \ldots & t_{1j}^{D_{1j}} & \ldots & t_{1m}^{D_{1m}}\\ \vdots & \vdots & \vdots & \vdots & \vdots \\ \vdots & \vdots & \vdots & \vdots & \vdots \\ \vdots & \vdots & \vdots & \vdots & \vdots \\ \vdots & \vdots & \vdots & \vdots & \vdots \\ t_{i1}^{D_{i1}} & \ldots & t_{ij}^{D_{ij}} & \ldots & t_{im}^{D_{im}}\\ \vdots & \vdots & \vdots & \vdots & \vdots \\ \vdots & \vdots & \vdots & \vdots & \vdots \\ \vdots & \vdots & \vdots & \vdots & \vdots \\ \vdots & \vdots & \vdots & \vdots & \vdots \\ t_{m1}^{D_{m1}} & \ldots & t_{mj}^{D_{mj}} & \ldots & t_{mm}^{D_{mm}} \end{array}\right]\;\begin{array}{cc} ⟶ & d_{1}=\sum_{i=j}^{m}t_{1j}^{D_{1j}}\\ \; & \;\\ \; & \;\\ \; & \;\\ \; & \;\\ ⟶ & d_{i}=\sum_{i=j}^{m}t_{1j}^{D_{1j}},d_{i}=\sum_{j=1}^{m}t_{ij}^{D_{ij}},\;i=1,\ldots .,m\\ \; & \;\\ \; & \;\\ \; & \;\\ \; & \;\\ ⟶ & d_{m}=\sum_{j=1}^{m}t_{mj}^{D_{mj}} \end{array},\\ T_{D}^{\alpha }\;=\;\left[\begin{array}{ccccc} \frac{t_{11}^{D_{11}}}{d_{1}} & \ldots & \frac{t_{1j}^{D_{1j}}}{d_{1}} & \ldots & \frac{t_{1m}^{D_{1m}}}{d_{1}}\\ \vdots & \vdots & \vdots & \vdots & \vdots \\ \frac{t_{m1}^{D_{m1}}}{d_{m}} & \ldots & \frac{t_{ij}^{D_{ij}}}{d_{i}} & \ldots & \frac{t_{im}^{D_{im}}}{d_{i}}\\ \vdots & \vdots & \vdots & \vdots & \vdots \\ \frac{t_{m1}^{D_{m1}}}{d_{m}} & \ldots & \frac{t_{mj}^{D_{mj}}}{d_{i}} & \ldots & \frac{t_{mm}^{D_{mm}}}{d_{im}} \end{array}\right]=\left[\begin{array}{ccccc} t_{D}^{\propto 11} & \ldots & t_{D}^{\propto 1j} & \ldots & t_{D}^{\propto 1n}\\ \vdots & \; & \vdots & \; & \vdots \\ t_{D}^{\propto i1} & \ldots & t_{D}^{\propto ij} & \ldots & t_{D}^{\propto in}\\ \vdots & \; & \vdots & \; & \vdots \\ t_{D}^{\propto n1} & \ldots & t_{D}^{\propto nj} & \ldots & t_{D}^{\propto nn} \end{array}\right]. \end{array}$$

**Step 6 .**

Normalization of the complete criteria matrix (**T**_**C**_^∝^)

To normalize *T*_*C*_, the sum of each row *T*_*C*_^*ij*^ is calculated and then, in*T*_*C*_^*ij*^, each element is divided by the sum of the elements of the corresponding row.

(7) $$\begin{array}{c} T_{C}^{\propto }=\begin{array}{c} D_{1}\\ \vdots \\ \vdots \\ \vdots \\ D_{i}\\ \vdots \\ \vdots \\ \vdots \\ D_{n}\\ C_{11}\\ C_{12}\\ C_{1_{m_{1}}}\\ \vdots \\ C_{i_{1}}\\ C_{i_{2}}\\ C_{i_{mi}}\\ \vdots \\ C_{n_{1}}\\ C_{n_{2}}\\ C_{nm_{m}} \end{array}\left[\begin{array}{ccccc} T_{c}^{\propto 11} & \ldots & T_{c}^{\propto 1j} & \ldots & T_{c}^{\propto 1n}\\ \vdots & \; & \vdots & \; & \vdots \\ \vdots & \; & \vdots & \; & \vdots \\ \vdots & \; & \vdots & \; & \vdots \\ T_{c}^{\propto i1} & \ldots & T_{c}^{\propto ij} & \ldots & T_{c}^{\propto in}\\ \vdots & \; & \vdots & \; & \vdots \\ \vdots & \; & \vdots & \; & \vdots \\ \vdots & \; & \vdots & \; & \vdots \\ T_{c}^{\propto n1} & \ldots & T_{c}^{\propto nj} & \ldots & T_{c}^{\propto nn} \end{array}\right], \end{array}$$

**Step 7 .**

Formation of an unbalanced *W* super matrix

In this step, the complete connection matrix is normalized, *T*_*C*_^∝^ is calculated, and the supermatrix *W* is got.

(8) $$\begin{array}{c} W=\left(T_{c}^{\propto }\right)=\begin{array}{c} D_{1}\\ \vdots \\ \vdots \\ \vdots \\ D_{i}\\ \vdots \\ \vdots \\ \vdots \\ D_{n}\\ C_{11}\\ C_{12}\\ C_{1_{m_{1}}}\\ \vdots \\ C_{i_{1}}\\ C_{i_{2}}\\ C_{i_{mi}}\\ \vdots \\ C_{n_{1}}\\ C_{n_{2}}\\ C_{nm_{m}} \end{array}\left[\begin{array}{ccccc} W^{11} & \ldots & W^{i1} & \ldots & W^{n1}\\ \vdots & \; & \vdots & \; & \vdots \\ \vdots & \; & \vdots & \; & \vdots \\ \vdots & \; & \vdots & \; & \vdots \\ W^{1j} & \ldots & W^{ij} & \ldots & W^{nj}\\ \vdots & \; & \vdots & \; & \vdots \\ \vdots & \; & \vdots & \; & \vdots \\ \vdots & \; & \vdots & \; & \vdots \\ W^{1n} & \ldots & W^{in} & \ldots & W^{nn} \end{array}\right], \end{array}$$

**Step 8 .**

Formation of a rhythmic supermatrix

To form a rhythm supermatrix, complete normal connection matrix *T*_*D*_^∝^ transpose and multiply by an unbalanced supermatrix.

(9) $$\begin{array}{c} W^{\propto }=T_{D}^{\propto }W=\left[\begin{array}{ccccc} t_{D}^{\propto 11}\times W^{11} & \ldots & t_{D}^{1i1}\times W^{i1} & \ldots & t_{D}^{\propto n1}\times W^{n1}\\ \vdots & \; & \vdots & \; & \vdots \\ t_{D}^{\propto 1j}\times W^{1j} & \ldots & t_{D}^{\propto ij}\times W^{ij} & \ldots & t_{D}^{\propto nj}\times W^{nj}\\ \vdots & \; & \vdots & \; & \vdots \\ t_{D}^{\propto 1n}\times W^{1n} & \ldots & t_{D}^{\propto in}\times W^{in} & \ldots & t_{D}^{\propto nn}\times W^{nn} \end{array}\right]. \end{array}$$

**Step 9 .**

Limit the rhythmic supermatrix

By powering a large number *Z*, until the supermatrix converges and stabilizes, the output of this step will be the effective DANP weights [27].

(10) $$\begin{array}{c} \underset{Z⟶\infty }{\lim}{\left(W^{\propto }\right)}^{Z}. \end{array}$$

### 2.3. Prioritize Water Resources in Floods

To prioritize Bandar Abbas water resources in floods, VIKOR technique with Excel software was utilized. The subcriteria were divided into two categories: quantitative and qualitative. Quantitative subcriteria were got from organization's information and studies, and qualitative criteria from a 9-point Likert scale and the opinions of 12 experts were utilized and summarized.

Opricovic proposed the VIKOR technique as one of the techniques relevant to MCDM. In situations where the decision-maker is not able to determine and express the advantages of a problem, this method can be considered an effective instrument for decision-making [28].

### 2.4. Steps of VIKOR Method

#### 2.4.1. Forming a Decision Matrix

According to the number of criteria, the number of options, and the evaluation of all options for different criteria, the decision matrix is formed as follows:

(11) $$\begin{array}{c} X=\left[\begin{array}{ccc} X_{11} & \cdots & X_{1n}\\ \vdots & \ddots & \vdots \\ x_{m1} & \cdots & X_{mn} \end{array}\right]. \end{array}$$

In that, *X*_*ij*_ is the function of option *i* about criterion *j*.

#### 2.4.2. Scaling the Decision Matrix

In this step, we try to convert the criteria with different dimensions into dimensionless criteria, and the *F* matrix is defined as follows:

(12) $$\begin{array}{c} f_{ij}=\frac{X_{ij}}{\sqrt{\sum_{i=1}^{n}X_{ij}^{2}}},\\ F=\left[\begin{array}{ccc} f_{11} & \cdots & f_{1n}\\ \vdots & \ddots & \vdots \\ f_{m1} & \cdots & f_{mn} \end{array}\right]. \end{array}$$

#### 2.4.3. Determining the Weight Vector of Criteria

The important factor of different criteria in decision-making is defined as follows:

(13) $$\begin{array}{c} W=\left[W_{1},W_{2},\ldots W_{n}\right]. \end{array}$$

#### 2.4.4. Determining the Best and Worst Value among the Available Values for Each Criterion

The best and worst values for the positive and negative criteria are calculated from the following equation:

(14) $$\begin{array}{c} f_{j}^{*}=Maxf_{ij},\\ f_{j}^{-}=M\mathrm{in}f_{ij}. \end{array}$$

#### 2.4.5. Calculating the Amount of Utility (*S*) and the Amount of Regret (*R*): These Values Are Calculated According to the Following Relations

(15) $$\begin{array}{c} R_{j}=\max\left\lceil W_{i}\cdot \frac{f_{j}^{*}-f_{ij}}{f_{j}^{*}-f_{i}^{-}\;}\right\rceil ,S_{j}=\sum_{i=1}^{n}W_{i}\cdot \frac{f_{j}^{*}-f_{ij}}{f_{j}^{*}-f_{i}^{-}\;}, \end{array}$$

where *W*_*j*_ is the desired weight value for criterion _j_.

#### 2.4.6. Calculating VIKOR *Q* Index: The Value of *Q* Is Calculated According to the Following Equation

(16) $$\begin{array}{c} Q_{i}=V\frac{S_{i}-S^{-}}{S^{*}-S^{-}}+\left(1\;-V\right)\left[\frac{R_{i}-R^{-}}{R^{*}-R^{-}}\right],\\ S^{-}=MinS_{i},S^{*}=MaxS_{i},\\ R^{-}=MinR_{i},R^{*}=MaxR_{i}. \end{array}$$

These relations express the distance rate from the ideal limit and *t* is from the counter-ideal limit, and parameter *V* is selected according to the agreement of the decision-making group.

#### 2.4.7. Ranking the Alternatives by Sorting *S*, *R*, and *Q* Values

Rank the alternative sorting by S, R, and Q values. Option A(1) as a compromise solution is suggested if the following two circumstances are satisfied:

- Acceptable advantage. *Q* ((A2)) _ *Q* ((A1)) ≥DQ, where DQ = 1/j-1; A(2) is the alternative with the second position in the ranking list by Q.
- Acceptable stability in decision-making. The alternative A(1) must also be the best ranked by *S* or/and *R*; this compromised solution is stable within a decision-making process, which could be the strategy of maximum group utility (when *v* > 0.5 is needed) or “by consensus” (*v*  > 0.5) or with veto (*v*  < 0.5).

If one of the conditions is not satisfied, then a set of compromised solutions can be proposed, including the following:

Alternatives A(1) and A(2) if only condition *b* is not satisfied.

Alternatives A(1), A(2)...A(*M*) if condition A is not satisfied. A(*M*) is determined by the relation *Q* (AM-A1) < DQ for maximum *M* (the positions of these alternatives are “in closeness”) [28].

## 3. Results

After reviewing and extracting the criteria and indicators from various studies, 9 main criteria and 44 subcriteria were defined to select water resources in disasters and emergencies. According to field studies and related organizations information, the proposed water resources for Bandar Abbas to use in flood are mentioned below.

### 3.1. Bandar Abbas Wastewater Treatment Plant Effluent

The amount of wastewater produced in Bandar Abbas is 70,560 cubic meters per day, of which 67,815 cubic meters per day is collected and treated by the Bandar Abbas wastewater treatment plant, and 1000 cubic meters per day by the treatment plants of the towns [29].

### 3.2. Humidity

The atmosphere holds 12,900 cubic kilometres of freshwater, of which 98 percent is in the form of steam and 2 percent in the form of clouds [30]. There are places on Earth where drinking water can be extracted from the atmosphere [31]. In Iran, especially in the southern coastal cities such as Bandar Abbas, the humidity in summer is very high and can be a drinking water resource [32].

### 3.3. Sea

The use of desalination technology is mainly in arid regions of the world, especially in the Middle East, where conventional freshwater resources such as rivers, lakes, or groundwater are not readily available. Technology has been very effective [33].

### 3.4. Sarkhoon Plain

Sarkhoon aquifer (7636 hectares) is approximately 30 kilometres from Bandar Abbas. This plain is one of the critical forbidden plains [34].

Table 1 shows the main criteria and subcriteria, quantitative and qualitative characteristics of water resources, and the weight of each subcriterion specified by the DANP technique in flood.

### 3.5. Prioritization of Water Resources

Table 2 shows the amount of *S*, *R*, and *Q* calculated based on the VIKOR technique and the rank of each proposed water resource.

Since the number of options is 4, DQ = 1/(J-1) = 1/(4-1) = 0.33 will result in Q ((A2)) _ *Q* ((A1)) = 0.128–0.0489 = 0.0791 ≥ 0.33.

Fewer *Q* values represent the optimal answer.

Because the above relation is not established, the condition of acceptable advantage is not established too. Therefore, based on the relation *Q* (AM-A1) <DQ, both effluent and sea options are the optimal answer. They also have a high rating in terms of *R* or *S* (acceptable stability condition).

For sensitivity analysis, it is necessary to change the value of *V* in the range of zero and one to examine the effect of the agreement coefficient on the result and the optimal answer.  Table 3 shows the sensitivity analysis based on the value of *V* in the range of zero and one.

To ensure that the results are valid or not, calculations were performed using the COPRAS method, and the results are showen as follows (higher *U* indicates optimal answer).  Table 4 shows the results of the COPRAS technique.

## 4. Discussion

Results showed that the optimal water resources for Bandar Abbas in flood disasters are the sea and wastewater treatment plant effluent (after treatment). Sensitivity analysis confirmed the results of appropriate water resource options. Also, the results of VIKOR (water resources prioritization) were confirmed by COPRAS method.

Membrane filtration systems, reverse osmosis, and seawater desalination for the sea source should be utilized to treat the proposed resources during floods. Also, to treat and use effluent of the Bandar Abbas wastewater treatment plant, membrane filters, nanofiltration, and advanced treatment are needed. In similar studies such as that by Qu [11], membrane filter technology, especially Ultrafiltration (UF), is utilized to treat saline and turbid water sources in emergencies. In Sadeghi Yekta's [13] study, the use of a “general desalination system” is suggested as the most suitable system for supply in semiarid regions facing severe water shortages. In Saiful's [15] study, the use of membrane filters and reverse osmosis system has identified the best and most appropriate method for water supply in emergencies. In Santos's [17] study, the use of membrane filters and *Moringa* determined the most suitable option for the point-of-use site water supply.

In this study, a combination of ANP and DEMATEL techniques is utilized for weighing the criteria. In the real world, relationships between decision criteria can have a network structure, so the problem cannot be solved with a hierarchical structure and linear methods such as AHP. Saaty [25] developed the Analytic Network Process (ANP) method to release the limitation of the linear techniques. Also, an unweighted supermatrix generated pairwise comparisons to calculate the weight of the significance of the dimensions/criteria. However, in the combined DANP method based on DEMATEL, the network structure and dimensions are determined by the DEMATEL, and, on the basis of the total effect matrix, the DEMATEL method is used to form an unweighted supermatrix for the ANP method. In this study, according to the network structure and internal and external dependence of the criteria and subcriteria obtained, the advantages of both methods in calculating weights have been used to adapt to more real-world problems.

 While in the studies of Sarband [45], Malek Mohammadi [14], Pagano [46], Ghandi [47], Amorim [14], Santos [17] AHP technique, Pagsuyoin [12], Loo [8] Decision Matrix Table, and Qu [11] the TFNs (Triangular Fuzzy Number) technique were used.

In this study, to prioritize the water resource options, the VIKOR technique was utilized. VIKOR technique is based on consensual planning of multicriteria decision-making. VIKOR assesses problems with disproportionate criteria. In cases where the decision-maker cannot identify and express the problem benefits at the time of its initiation and design, this method can be considered an effective instrument for decision-making.

The VIKOR method also has excellent features that other multicriteria decision-making methods such as TOPSIS, SAW, and COPRAS do not have. This method has been developed for multicriteria optimization of complex systems. This method focuses on categorizing and selecting from a set of options and determines compromising solutions to a problem with conflicting criteria. Here the compromised answer is the closest justified answer to the ideal solution. The word compromise refers to a mutual agreement. The VIKOR method uses an aggregate function that expresses the distance from the ideal solution. This ranking index is a sum of all the criteria, the relative importance of the criterion, and a balance between majority satisfaction and individual satisfaction. On the other hand, the values normalized in the VIKOR method do not depend on the evaluation unit of each criterion because it uses linear normalization. Therefore, in this study, the VIKOR technique was used to prioritize the alternatives [28].

While in studies of Sarband [45] Distributed Spatial Indices with ANP technique, Ghandi [47], Fuzzy PROMETHEE V technique, Santos [17], Pagsuyoin [12], Qu[11], TOPSIS technique, and Sadeghi Yekta [13] Distance-Based Fuzzy Multi-Criteria Group Decision Making technique (DBF-MCDM) were used.

The most significant criteria with the highest weight in the flood were the treatment degree (0.0834), population density (0.0492), health compatibility (0.0413), community acceptance (0.0397), and complexity level (0.0327). The least significant criteria with the lowest weight in flood were humidity (0.0001), land use (0.0001), region climate (0.0001), annual rainfall (0.0001), and easy access to roads (0.0063).

## 5. Conclusion

Floods are the most important natural disasters that cause great damage, especially to infrastructures, including drinking water resources. Drinking water supply is one of the most basic needs after disasters. Using water resources in disaster-prone areas is more stable and practical, so, in this study, available water resources for flood disasters drinking water supply in Bandar Abbas were identified (sea, humidity, Sarkhon plain, and effluent). After weighing the criteria with the DANP technique and prioritizing water resources with the VIKOR technique, sea and wastewater treatment plant effluent (after advanced treatment) were recognized as water resources supply for use in Bandar Abbas flood disasters. The study proposed appropriate model to select optimal water resources for various natural disasters in different geographical areas. This model can help officials and decision-makers to plan for drinking water supply from disaster-prone areas before disasters occur.

## Figures and Tables

**Figure 1:** Flow diagram of the study method.

**Table 1:** Main criteria and subcriteria, quantitative and qualitative characteristics of water resources, and the weight of each subcriterion in flood.

Main criteria	Subcriteria	Qualitative/quantitative	Unit	Aspect	Effluent	Sea	Air humidity	Sarkhoon plain	Weight
Environmental factors	Toxicity of by-products	Qualitative	—	Negative	7	7	1	3	0.032
	Health compatibility	Qualitative	—	Positive	5	5	6	6	0.0413
	Community acceptance	Qualitative	—	Positive	3	6	6	6	0.0397
Economic factors	Equipment cost	Qualitative	—	Negative	8	8	7	2	0.0295
	Construction cost	Qualitative	—	Negative	8	7	6	3	0.0295
	Operating and maintenance costs	Qualitative	—	Negative	9	8	7	3	0.0293
	Material cost	Qualitative	—	Negative	9	7	6	3	0.0289
Regional geographical factors	Humidity	Qualitative	—	Positive	3	1	9	6	0.0001
	Population density	Qualitative	—	Negative	5	2	2	6	0.0492
	Annual rainfall	Qualitative	—	Positive	6	2	7	8	0.0001
	Land use	Qualitative	—	Negative	7	4	3	7	0.0001
	Region climate	Qualitative	—	Negative	4	5	8	6	0.0001
General characteristics of water treatment system	Ease of deployment	Qualitative	—	Positive	2	3	4	5	0.0311
	Complexity level	Qualitative	—	Negative	9	7	7	4	0.0327
	Ease of use	Qualitative	—	Positive	1	4	4	6	0.0319
	Supply chain needs	Qualitative	—	Negative	9	7	6	3	0.0321
Technical characteristics of water treatment systems	Production capacity	Quantitative	m^3^/d	Positive	10 [29]	10000 [35]	40 [36]	3000 [37]	0.0237
	Energy consumption	Quantitative	Kw/m^3^	Negative	224.39 [26]	8 [37]	292 [36]	0.0682 [37]	0.0233
	Heavy metals removal	Quantitative	%	Positive	95 [29]	90 [37]	0 [36]	0 [29]	0.0147
	Performance efficiency	Qualitative	—	Positive	7	6	6	4	0.0232
	Operation and maintenance	Qualitative	—	Negative	9	8	7	4	0.0227
	Technical maturity	Qualitative	—	Positive	1	5	5	7	0.0219
General characteristics of water resources	Distance to residential areas	Quantitative	km	Negative	1 [29]	1 [29]	0.00001 [29]	30 [29]	0.0095
	Distance to pollutant sources	Quantitative	km	Positive	15 [29]	15 [29]	15 [29]	10 [29]	0.0095
	Water source capacity	Quantitative	m^3^/d	Positive	67815 [29]	1000000 [38]	221392 [39]	4928000 [34]	0.0086
	Treatment degree	Qualitative	—	Negative	9	7	4	4	0.0833
	Easy access to roads	Qualitative	—	Positive	6	6	8	5	0.0063
Nontoxic chemicals of water sources	Nitrate	Quantitative	mg/l	Negative	7.67 [29]	0.0182 [40]	0.06 [36]	19.7 [41]	0.0202
	Total hardness	Quantitative	mg/l	Negative	344.55 [29]	4975.79 [35]	38.81 [42]	389.6 [41]	0.0194
	Sodium	Quantitative	mg/l	Negative	6.45 [29]	9715 [41]	0.069 [43]	115.2 [41]	0.0153
	Chloride	Quantitative	mg/l	Negative	118 [29]	20109.5 [35]	3.5 [36]	156 [41]	0.0153
	Sulfate	Quantitative	mg/l	Negative	261.3 [29]	2491.4 [35]	0.1 [43]	248 [41]	0.0153
	Calcium	Quantitative	mg/l	Negative	33.9 [29]	416 [44]	0.176 [43]	93.9 [41]	0.0153
	Magnesium	Quantitative	mg/l	Negative	31 [29]	1581 [44]	0.0355 [43]	37.2 [41]	0.0153
Toxic chemicals of water sources	Mercury	Quantitative	mg/l	Negative	0.0001 [29]	0.011 [38]	0.001 [43]	0.0001 [41]	0.0283
	Lead	Quantitative	mg/l	Negative	0.133 [29]	10.36 [38]	0.001 [43]	0.003 [41]	0.0283
	Chrome	Quantitative	mg/l	Negative	0.012 [29]	98.8 [38]	0.001 [43]	0.00001 [41]	0.0283
	Cadmium	Quantitative	mg/l	Negative	0.0054 [29]	0.17 [38]	0.001 [43]	0.009 [41]	0.0283
Physical and biological characteristics of water resources	pH	Quantitative	—	Negative	7.38 [29]	8.1 [40]	6.81 [42]	7.6 [41]	0.0188
	Turbidity	Quantitative	NTU	Negative	40.7 [29]	70.7 [40]	2.4 [42]	0.46 [41]	0.0178
	TDS	Quantitative	mg/l	Negative	1687.1 [29]	43400 [40]	31.7 [42]	778.8 [41]	0.0207
	Electrical conductivity	Quantitative	µm/cm	Negative	5970 [29]	57000 [40]	42.54 [42]	1298 [41]	0.0207
	Total coliform	Quantitative	MPN	Negative	1220 [29]	2393.45 [29]	16.5 [42]	10 [41]	0.0192
	Fecal coliforms	Quantitative	MPN	Negative	430 [29]	800.4 [29]	6.03 [42]	4 [41]	0.0192

**Table 2:** Ranking of proposed water resources.

V = 0.5	Effluent	Sea	Air humidity	Sarkhoon plain
S	0.254392709	0.213518839	0.547656646	0.524223508
R	0.0413	0.0492	0.0833	0.0833
Q	0.061163194	0.094047619	1	0.964934919
Rank	1	2	4	3

**Table 3:** The results of sensitivity analysis.

*V* = 0.1	Effluent	Sea	Air humidity	Sarkhoon plain
* S*	0.254392709	0.213518839	0.547656646	0.524223508
* R*	0.0413	0.0492	0.0833	0.0833
* Q*	0.012232639	0.169285714	1	0.992986984
Rank	1	2	4	3
*V* = **0.2**				
* S*	0.254392709	0.213518839	0.547656646	0.524223508
* R*	0.0413	0.0492	0.0833	0.0833
* Q*	0.024465277	0.15047619	1	0.985973968
Rank	1	2	4	3
*V* = **0.3**				
* S*	0.254392709	0.213518839	0.547656646	0.524223508
* R*	0.0413	0.0492	0.0833	0.0833
* Q*	0.036697916	0.131666667	1	0.978960951
Rank	1	2	4	3
*V* = **0.4**				
* S*	0.254392709	0.213518839	0.547656646	0.524223508
* R*	0.0413	0.0492	0.0833	0.0833
* Q*	0.048930555	0.112857143	1	0.971947935
Rank	1	2	4	3
*V* = **0.6**				
* S*	0.254392709	0.213518839	0.547656646	0.524223508
* R*	0.0413	0.0492	0.0833	0.0833
* Q*	0.073395832	0.075238095	1	0.957921903
Rank	1	2	4	3
*V* = **0.7**				
*S*	0.254392709	0.213518839	0.547656646	0.524223508
* R*	0.0413	0.0492	0.0833	0.0833
* Q*	0.085628471	0.056428571	1	0.950908886
Rank	2	1	4	3
*V* = **0.8**				
* S*	0.254392709	0.213518839	0.547656646	0.524223508
* R*	0.0413	0.0492	0.0833	0.0833
* Q*	0.09786111	0.037619048	1	0.94389587
Rank	2	1	4	3
*V* = **0.9**				
* S*	0.254392709	0.213518839	0.547656646	0.524223508
* R*	0.0413	0.0492	0.0833	0.0833
* Q*	0.110093749	0.018809524	1	0.936882854
Rank	2	1	4	3

**Table 4:** The results of COPRAS technique.

	Effluent	Sea	Air humidity	Sarkhoon plain
*Q*_*i*_	0.665889756	0.654010972	0.368866505	0.413487597
*U*_*i*_	1	0.982161035	0.553945308	0.620955035
***U***_***i***_ ^*∗*^**100**	100	98.21610354	55.39453075	62.09550355
Rank	1	2	4	3

## Data Availability

The data used to support the findings of this study are included within the article.
